The article "Deducing Leading Factors of Spatial Distribution of Carbon Reserves in Nanjing Metropolitan Area Based on Random Forest Model" was published in 2022. Journal: Comput Intell Neurosci.

# Deducing Leading Factors of Spatial Distribution of Carbon Reserves in Nanjing Metropolitan Area Based on Random Forest Model

**DOI:** 10.1155/2022/3013620

**Published:** 2022-08-25

**Authors:** Jiefu Xue, Jun Yan

**Affiliations:** College of Landscape Architecture, Nanjing Forestry University, No. 159 Longpan Road, Nanjing 210037, Jiangsu, China

## Abstract

Improving carbon reserves is considered to be an important way to alleviate global warming. However, there is a lack of research work based on the perspective of metropolitan area, and there is also a lack of analysis on the leading influencing factors of spatial distribution of carbon storage in subregions of metropolitan area. In this study, Nanjing metropolitan area (NMA) is taken as the research area, and the InVEST model is used to calculate the spatial distribution of regional carbon reserves, and the evolution of carbon reserves distribution in recent 20 years is analyzed. Then, based on the random forest (RF) model, taking the whole study area and subareas as the research scope, a regression model of each selected impact factor and carbon reserves is established, and the leading factors of spatial distribution of carbon reserves in NMA are obtained. The results show that the overall carbon reserves level in the study area is in a downward trend. Through the application of the RF model, the leading factors of the spatial distribution of carbon reserves in NMA and its subareas are derived. The research proves that the application of the RF model in the analysis is helpful for city planners and governments to make plans and improve regional carbon storage more effectively.

## 1. Introduction

Global warming is an international challenge that all mankind needs to face in the twenty-first century [1]. To meet this challenge, China will strive to achieve peak carbon dioxide emissions by 2030 and carbon neutrality by 2060. Carbon reserves are widely regarded as an important indicator of ecosystem services [2]. Carbon stored in terrestrial ecosystems plays a very important role in global carbon cycle, atmospheric carbon dioxide concentration, and global climate change. Terrestrial ecosystems capture greenhouse gases such as CO_2_ and CH_4_ through forests, grasslands, and other green infrastructure to regulate the regional climate and increase the carbon reserves [3].

Since 1850, changes of LULC have caused the global terrestrial ecosystem to lose 145 Pg C [4]. Therefore, quantitative analysis and prediction of ecosystem carbon reserves based on LULC plays an important role in achieving carbon neutrality, improving global climate, and fully protecting the ecosystem. Cities are the areas with the most transformation, the fastest change rate, and the most frequent land use activities in the urban terrestrial ecosystem [5]. With the rapid development of industry, cities have become the main areas where chemical fuels are burned, and more than 80% of CO_2_ emissions come from cities [6, 7]. Urban carbon reserves have become an important factor affecting the regional climate and regional ecosystem.

At present, the methods used to study the carbon reserves at home and abroad mainly include biomass method [8, 9], bookkeeping method [10], and inventories method of the Intergovernmental Panel on Climate Change (IPCC) [11, 12]. In recent years, most scholars began to use the *Integrated Valuation of Ecosystem Services and Trade-off*s (InVEST) model, which runs fast, requires less data, and is practical, to study the carbon reserves in watersheds [13, 14], cities [15–17], special geographical area [18], and other areas. Those points out that the study of carbon reserves has important reference value for the management of terrestrial ecosystem carbon pool.

With the deepening of China's urbanization process, the development of Chinese cities has shifted from focusing on each city's own urbanization to focusing on interregional cooperation and development among different cities [19, 20]. There have been examples of establishing large metropolitan areas across municipal or even provincial administrative regions. At present, the academic research on urban carbon reserves mainly focuses on the change of carbon reserves based on LULC change [21–24]. Some studies analyzed the evolution of historical LULC in the region, and used some simulation models such as CA-Markov to predict the LULC change in multiple scenarios in the future, so as to deduce the future change trend of regional carbon reserves [25–27]. Those studies have achieved fruitful results in solving the corresponding research issues, but there is still a lack of analysis and research work based on the perspective of metropolitan area, as well as the analysis of the leading influencing factors of spatial distribution of carbon reserves in subregions at all levels in the metropolitan area.

The random forest (RF) model is an ensemble learning algorithm [28, 29], which aggregates multiple classification trees, and each tree is assigned by random vectors sampled independently. Among the existing algorithms, the RF algorithm has good accuracy and can be effectively run on large data sets [29, 30]. It can be used to assess the importance of each feature in the classification [31]. While using RF model, researchers do not need to worry about the problem of multicollinearity. At the same time, RF model can calculate the nonlinear interaction between variables and reflect the interaction between them [32]. Besides, RF model are not sensitive to outliers [29]. It has shown amazing performance on classification and regression issues. Compared with the other methods, the random forest is suitable for processing high-dimensional data, is not easy to generate overfitting, and performs well when processing the data [31, 33, 34]. At present, RF model has been widely used in medicine [35, 36], economics [37, 38], remote sense [39, 40], and some other fields, but it has not been widely used in the research of carbon reserves.

To sum up, we select Nanjing metropolitan area (NMA), the first national metropolitan area in China, as the research area. We calculate the regional carbon reserves spatial distribution by using the InVEST model, and verify and analyze the evolution of carbon reserves distribution in the past 20 years (2000–2020). The core of our work is to establish the regression model of each influencing factor and carbon reserves based on the RF model, and obtain the leading factors of spatial distribution of carbon reserves in NMA, in order to provide the basis for realizing carbon neutralization, improving the carbon reserves capacity of the ecosystem, and reasonably formulating the land use strategy in NMA.

## 2. Material and Methods

### 2.1. Study Area and Data Collection

Nanjing Metropolitan Area (NMA) is the first planned national metropolitan area in China (Figure 1). NMA is in the core area of the urban belt along the Yangtze River in eastern China, spanning Jiangsu and Anhui provinces. NMA includes Nanjing City, Zhenjiang City, Yangzhou City, Huai'an City, Ma'anshan City, Chuzhou City, Wuhu City, Xuancheng City, Liyang City, and Jintan County in Changzhou City. It includes 33 municipal districts, 11 county-level cities, and 16 counties, with a total area of 66,000 square kilometers. Located in the alluvial plain formed by humid monsoon climate in East China, NMA belongs to the humid area in the north subtropical zone. The regional vegetation belongs to the mixed forest of deciduous and evergreen broad-leaved vegetation in the northern subtropical zone. The key service function of this area is urban ecology. However, with the unlimited expansion of cities and metropolitan areas, the ecological carrying capacity of NMA is seriously overloaded, the ecological functions are reducing, the pollution is serious, and the quality of human settlements is reduced [41–43].

NMA involves a number of different administrative divisions belonging to different provinces, and the regional scale is large, and the economic volume, ecological environment, and other factors of each constituent city are very different. Therefore, we not only explore the influencing factors of carbon reserves change in NMA, but also explore the differences of those factors in different subareas of NMA. Generally speaking, the planning of administrative regions at all levels in China is mostly based on the county level or above (county is city's next administrative unit, Xi'an or Qu in Chinese). Taking each county-level region in NMA as a unit and combining with the development plan of NMA published by the National Development and Reform Commission of China, the research area is divided into three subareas: urban core area (UCA), urban planning area (UPA), and urban expansion area (UEA).  Table 1 lists the county-level administrative regions included in the study area and subareas.

All the data used in the thesis are projected and resampled in ArcGIS software before further processing. The data describing the spatial distribution characteristics of annual precipitation come from the National Earth System Science Data Center (https://www.geodata.cn) of China's national science and technology infrastructure. The extracted images of elevation and slope are from GDEM·V2 of Land Processing Distributed Activity Archive Center (LP DAAC) of NASA. Normalized Difference Vegetation Index (NDVI) data is calculated by using 59 Landsat-8 remote sensing images taken in 2020. Potential evapotranspiration, average temperature, road network, railways network, population, and urban water system data are from the Data Center of Resources and Environmental Sciences, Chinese Academy of Sciences (https://www.resdc.cn/).

### 2.2. Study Design

This thesis can be divided into the following three steps:

  First, taking Nanjing Metropolitan Area (NMA) as the research area, the spatial distribution of regional carbon reserves is calculated by using the carbon module of InVEST model, and the evolution of carbon reserves distribution in recent 20 years (2000–2020) is analyzed.
  Second, we select the land use types and the driving factors of land use evolution required for the research as the influencing factors adopted in the research.
  Third, based on the RF model, the regression models of various influencing factors and carbon reserves are established for the whole study area and each subarea to obtain the dominant factors of NMA carbon reserves spatial distribution.

### 2.3. Calculation and Evolution Analysis of Carbon Reserves Based on InVEST Model

This paper discusses the regional evolution trend of carbon reserves in NMA based on InVEST model. We calculate the spatial and temporal distribution of Carbon reserves in NMA from 2000 to 2020 using the Carbon module of InVEST model. The carbon reserves calculated by Carbon module include four carbon pools, i.e., aboveground biomass carbon pool, underground biomass carbon pool, soil carbon pool, and dead organic matter carbon pool. The calculation formula of carbon reserves is as follows [15]:

(1) $$\begin{array}{c} C_{\text{total}}=C_{\text{above}}+C_{\text{below}}+C_{\text{soil}}+C_{\text{dead}}, \end{array}$$

where *C*_total_ is the regional total carbon reserves, *C*_above_ is the aboveground biomass carbon reserves, *C*_*below*_ is the underground biomass carbon reserves, *C*_*soil*_ is the soil carbon reserves, and *C*_*de*  *a*  *d*_ is the dead organic matter carbon reserves (*t*/*km*^2^).

Carbon reserves is affected by factors such as location, altitude, hydrothermal condition, and land use, which leads to differences in carbon sequestration characteristics in different regions, thus affecting terrestrial ecosystems [31, 44]. The values of carbon density in the study area are quoted from the calculation results of Chinese scholar Liu and Zhu [45], etc., as shown in Table 2.

Based on the above, combined with the LULC in 2000, 2010, and 2020, we can obtain the carbon reserves distribution of NMA in the corresponding years. Then, according to the principle of equal interval, the distribution of carbon reserves in NMA obtained in the previous steps is divided into level A, B, C, and D from low to high, and the proportion of the four levels in each year is calculated, respectively. Finally, the carbon reserves data of adjacent years are subtracted to get the change of carbon reserves every 10 years.

### 2.4. Deducing of Leading Factors of Carbon Reserves in NMA Based on RF Model

The distribution of regional carbon reserves is influenced by many factors, which are the result of the interaction of physical and chemical conditions of various types of land and various factors such as nature and society [31, 44]. The impact of land use change on regional carbon reserves is very prominent, and the driving factors of land use change can also affect the spatial and temporal changes of regional carbon reserves [46]. Therefore, in this study, various land use types and commonly used driving factors of land use evolution are used to infer and analyze the driving factors of carbon reserves evolution. The driving factors selected in this study include DEM (elevation), SLOPE, TEM (temperature), PRE (precipitation), PET (potential evapotranspiration), RRO_ROAD (proximity to roads), RRO_RAIL (proximity to railways), POP (population), GDP (Gross Domestic Product), RRO_WATER (proximity to water bodies), FOREST COVERAGE, and LULC. The data sources of DEM, TEM, PRE, PET, GDP, and POP have been given above. SLOPE is calculated from DEM data in ArcGIS using the slope calculation tool in the surface analysis module and FOREST COVERAGE is obtained by converting NDVI data of Nanjing for the whole year of 2020. RRO_WATER and RRO_ROAD are calculated by applying Euclidean distance tool to the corresponding data. The impact factors are shown in Figure 2.

According to the scale of the study area and the actual situation of the required data, a sampling surface with a unit grid of 3 × 3 km was set up in NMA by using ArcGIS software, and the grid data including carbon reserves distribution and various influencing factors are sampled. On this basis, taking the carbon reserves of NMA in 2020 as dependent variable and various land use types and driving factors as independent variable, the RF model is used to deduce and analyze the leading factors of carbon reserves' distribution.

The random forest algorithm is a combination classification algorithm proposed by Breiman [28], and it is a supervised learning algorithm that integrates multiple decision trees [28, 35]. It is often used for classification and regression in machine learning. Classification and regression can be completed based on the data processing results. Its working principle is to build multiple decision trees in a given training time, and output the model as the class (classification) or average prediction (regression) of each tree. The core of the RF model is the binary tree model finally generated by CART [28]. Error estimation and tree pruning are carried out by using the recapture technology, and the best model is selected as the final decision tree.

In the process of learning and training of RF, data are generally divided into training set and test set for modeling and simulation (prediction) [33]. Firstly, the training set is used for training and learning, and the optimal parameters are found. Secondly, the test set is used to evaluate the actual performance of the model learned from the training data set. The selection of training samples and test samples is the precondition of modeling random forest.  Figure 3 is a framework of the principle of RF model in regression analysis.

In this study, the RF model is constructed by using the extracted related variables. According to the method of modeling, the data (feature) sample set is divided into two parts: training set (70% of the total) and test set (30% of the total). The error and goodness-of-fit (*R*^2^, coefficient of determination) between the predicted values and actual values of test set are analyzed. Generally speaking, if the *R*^2^ of the model is greater than 0.8, the model can be considered as meeting the requirements. After the running of the model, we can get the order of the characteristic importance of each influencing factor, so as to get the leading factors of carbon reserves distribution.

## 3. Results and Discussion

### 3.1. Analysis on the Distribution and Evolution of Carbon Reserves in NMA

Figure 4 shows the spatial distribution of carbon reserves in NMA based on the InVEST model. It can be seen from the figure that rivers, lakes, and urban built-up areas are carbon reserves depressions. Taken together, the overall carbon reserves of the study area decreased obviously, which reflects the trend of outward expansion centered on the built-up areas of various administrative regions.  Table 3 shows the statistics of carbon reserves evolution of each level in NMA. It can be found that the region with the lowest carbon reserves grade expanded significantly, from 9.52% in 2000 to 13.85% in 2020. The area proportions of the two middle carbon reserves levels both decreased, while the proportion of the region with the highest grade increased slightly, from 9.54% in 2000 to 10.11%.

The distribution of regional carbon reserves change values can be seen from Figure 5. In combination with Figure 5 and Table 3, the change rate of carbon reserves is faster in the first decade (2000–2010) than in the second decade (2010–2020). The first decade corresponds to the so called “golden decade” of China's urban development. During this period, China's major cities are in a period of rapid expansion, focusing on the development of urban scale [19, 47]. The change in the second decade reflects that China has begun to pay attention to solving urban ecological problems and intends to control the speed of urban expansion [48]. The characteristics of urban development have changed from extensive expansion to refined urban details and infrastructure construction.

In summary, the development of cities has reduced the regional carbon reserves, although the planning work of some regions has emphasized the ecological restoration, objectively improved the carbon reserves level of the regions. However, minor repairs in some regions cannot reverse the decline in urban carbon reserves. In addition, the pace of urbanization cannot be stopped, so it is impossible to achieve the goal of promoting regional carbon neutrality by limiting the urban development. Therefore, it is urgent to analyze the metropolitan area and all levels of subareas to obtain the leading influencing factors of the spatial distribution of carbon reserves as planning's support, so as to make reasonable planning and arrangement for the spatial elements of all levels of regions in order to achieve the goal of carbon neutrality.

### 3.2. Leading Factors of Carbon Reserves Distribution in NMA Based on RF Model

Models established for NMA, UCA, UPA, and UEA are designated as model I, II, III, IV, and IV, respectively. According to the established RF model [49–58], the *R*^2^ of each level can be calculated. The numb of ntree is set as 100 as a parameter input.  Table 4 shows the errors and *R*^2^ of the RF model for NMA and its three subareas. From the table, *R*^2^ values of each model test set are well above 0.75.  Figure 6 shows the comparison between the predicted and actual values of the simulation predictions, and the prediction accuracy is good overall. In summary, the overall performance of the model is good, and the prediction ability is better, which indicates that the RF model has good application effect in NMA.

The importance ranking of factors obtained from the operation of the RF model is shown in Figure 7. It can be seen from the figure that the relative importance of the corresponding impact factors in each area is not the same, indicating that it is very necessary to carry out internal segmentation and further analysis of the metropolitan area. The importance of the sixteen factors is different, and the relative influence has a very wide gap. Therefore, the factors whose characteristic importance is less than 5% are not listed in this thesis. It can be seen from the figure that the importance of each factor in the whole area of NMA ranged from large to small is *x*_16_ > *x*_02_ > *x*_14_ > *x*_11_, that in the UCA ranged from large to small is *x*_11_ > *x*_13_ > *x*_14_ > *x*_16_, that in the UPA ranged from large to small is *x*_16_ > *x*_14_ > *x*_11_ > *x*_13_, and that in the UEA ranged from large to small is *x*_16_ > *x*_02_ > *x*_14_.

For NMA, LULC_Water bodies, slope, vegetation coverage, and LULC_Artificial surfaces are the main leading factors, of which LULC_Water bodies account for almost half (42.80%) and is the most important factor affecting the distribution of carbon reserves in NMA. NMA is located in the middle and lower reaches of the Yangtze River with abundant rainfall. There are a large number of lakes in the area, among which Xuanwu Lake and Gucheng Lake of Nanjing City, Gaoyou Lake of Yangzhou City, Hongze Lake of Huai'an City have relatively large water scales, which directly affects the regional carbon reserves distribution. In urban areas, the vegetation coverage is better in the areas with larger slope, such as Mount Zijin, Mount Niushou, and Mount Lao, where the carbon sequestration is relatively higher. For UCA, vegetation coverage, LULC_Cultivated lands, LULC_Artificial surfaces, and LULC_Water bodies are the leading factors, of which, vegetation coverage has the largest effect (64.10%) and contributes more than half. The UCA has a high degree of urbanization and is the core functional area of NMA. The artificial surfaces account for the largest proportion, and human activities have the most profound impact on the surface cover. The most important source of carbon reserves in this area is the vegetation. Compared with forests, the vegetation coverage derived from NDVI can better reflect the regional vegetation cover, and has a stronger explanation power for the regional carbon reserves distribution. For UPA, LULC_Water bodies, LULC_Artificial surfaces, vegetation coverage, and LULC_Cultivated lands are the leading factors that dominate the distribution of carbon reserves in the region, of which LULC_Water bodies, LULC_Artificial surfaces, and vegetation coverage have the similar explanatory power (28.30%, 20.60%, and 20.30%), with the comprehensive impact rate exceeding half. A large number of lakes are distributed in the UPA, and the urban development in the region cannot be underestimated. At the same time, the forest coverage is better than that of UCA. Therefore, the contribution to the distribution of carbon reserves is higher than that to UCA. For UEA, LULC_Water bodies, slope, and LULC_Artificial surfaces are the leading factors affecting the spatial distribution of regional carbon reserves, of which the contribution of LULC_Water bodies is more than half (54.40%). The urbanization rate of UEA is in the relatively lowest position in NMA, and the area distribution of water bodies involved in the region is relatively larger, such as part of Hongze Lake. In addition, a large number of mountains with good coverage of associated vegetation directly affected the regional carbon sequestration and carbon reserves distribution.

### 3.3. Limitations and Further Research

This paper provides a new idea for the study on the influencing factors of the spatial distribution of regional carbon reserves, and the indexes system adopted can provide a reference for the study of urban carbon reserves. This paper can help landscape and urban planners planning, but also has some limitations.

First, InVEST model can be used to evaluate ecosystem services at different scales, and the evaluation results can be displayed visually. However, the evaluation results of this model are greatly affected by the land use classification. For example, in this study, land use types are divided into six categories, and each land use type is assumed to be homogeneous internally, so the model lacks consideration of regional internal heterogeneity. In addition, the differences in economic development of different sites and different metropolitan areas may lead to the nonuniversality of the evaluation indexes system. Therefore, it is necessary to establish the different models to evaluate different regions of different cities, which needs to be considered in further research. At the same time, because the InVEST model is based on land use, factors other than land use may be overlooked in the analysis.

Firstly, in future research, we can model different types of cities and evaluate them according to local conditions. Secondly, it can take more cities as the research object, and the commonness and difference between each category can be analyzed at the same time, thus proposing a more universal evaluation indexes system, determining the commonness problems between cities according to the regression analysis results, and proposing a more universal planning strategy. Thirdly, we can list other influencing factors except land use in the follow-up research, so as to carry out analysis and discussion. At the same time, as a holistic and systematic project, carbon reserves research should be actively integrated into related disciplines to promote the overall cooperation among different disciplines.

## 4. Conclusion

In this study, Nanjing metropolitan area (NMA) was taken as the study area, and the Carbon module of InVEST model was used to calculate the spatial distribution of regional carbon reserves, and the evolution of carbon reserves distribution in recent 20 years was analyzed. Then, based on the random forest (RF) model, taking the whole study area and subregions at all levels as the research scope, a regression model of each influencing factor and carbon reserves is established, and the leading factors of spatial distribution of carbon reserves in NMA were derived.

The results show that the overall carbon reserves in the study area is in a downward trend. The leading factors of the whole study area are LULC_Water bodies, slope, vegetation coverage, and LULC_Artificial surfaces, among which the influence of LULC_Water bodies is the most obvious. The leading factors of urban core area are vegetation coverage, LULC_Cultivated lands, LULC_Artificial surfaces, and LULC_Water bodies, among which the vegetation coverage contributes the most. The leading factors of urban planning area include LULC_Water bodies, LULC_Artificial surfaces, vegetation coverage, and LULC_Cultivated lands, among which the explanatory power of LULC_Water bodies, LULC_Artificial surfaces, and vegetation coverage is similar, and the combined contribution offers more than half. The leading factors of urban expansion area include LULC_Water bodies, slope, and LULC_Artificial surfaces, among which LULC_Water bodies is the most important one.

Based on the results of the RF model, we can get the order of the characteristic importance of factors, thus providing the basis for decision-making. According to the research results and the above analysis, we can put forward the direction of NMA and the planning of each subareas, especially in the context of the increasingly prosperous carbon trading market. How to improve the regional carbon reserves more efficiently in urban planning, the RF model can have more room to play its role.

## Figures and Tables

**Figure 1:** Location of the study site.

**Figure 2:** Impact factors used in this thesis.

**Figure 3:** Framework of the RF model in this thesis.

**Figure 4:** Distribution of carbon reserves in NMA from 2000 to 2020.

**Figure 5:** Carbon reserves variation in 2000 to 2010 and 2010 to 2020.

**Figure 6:** Test set prediction results. (a) Test set prediction results of MODEL I (b) test set prediction results of MODEL II (c) test set prediction results of MODEL III (d) test set prediction results of MODEL IV.

**Figure 7:** The relative importance of the factors.

**Table 1:** Administrative regions included in the study area and subareas.

Area	Including administrative divisions
NMA	Nanjing metropolitan area
UCA	Nanjing city
UPA	Jingkou district, Runzhou district, Dantu district and Jurong city in Zhenjiang city, Guangling district, Hanjiang district, Jiangdu district and Yizheng city in Yangzhou city, Xuyi county in Huai'an city, Jinghu district, Yijiang district and Jiujiang district in Wuhu city, Anhui province, Huashan district, Yushan district, Bowang district, He county and Dangtu county in Ma'anshan city, Langya district and Nanqiao district in Chuzhou city
UEA	The areas except the above areas in Zhenjiang city, Yangzhou city, Huai'an city, Wuhu city, Maanshan city, Chuzhou city and Xuancheng city, and Jintan city and Liyang city in Changzhou city

**Table 2:** Carbon density of different LULC types used in this study.

Land use types	Carbon density (kg/m^3^)			
	Aboveground	Underground	Soil	Dead
Cultivated lands	1.8873	1.2457	8.6759	0.2410
Forests	3.6339	0.7268	12.0758	0.3354
Grasslands	1.7374	2.0849	10.5847	0.2940
Water bodies	0.0000	0.0000	8.1100	0.0000
Artificial surfaces	1.6153	0.3231	7.2920	0.0000
Bare lands	2.4291	0.4858	8.0719	0.2242

**Table 3:** Carbon reserves data of different levels in Nanjing metropolitan area.

Year		2000	2010	2020
Total area and proportion of each level	Level A	6230.3391	8101.602	9067.167
		9.52%	12.38%	13.85%
	Level B	47701.1169	45640.1502	44697.575
		72.88%	69.73%	68.29%
	Level C	5278.218	5084.54	5063.052
		8.06%	7.77%	7.74%
	Level D	6241.9599	6625.6569	6618.222
		9.54%	10.12%	10.11%

**Table 4:** The errors and *R*^2^ of the RF model for NMA and its subareas.

Area	Model	Set type	RMSE	MAE	MAPE	*R * ^2^
NMA	I	Training set	0.309	0.176	1.628	0.926
		Test set	0.377	0.207	1.905	0.892

UCA	II	Training set	0.123	0.089	0.886	0.982
		Test set	0.257	0.155	1.596	0.919

UPA	III	Training set	0.466	0.136	1.206	0.901
		Test set	0.348	0.171	1.586	0.884

UEA	IV	Training set	0.328	0.191	1.727	0.925
		Test set	0.412	0.226	2.036	0.888

## Data Availability

The dataset can be accessed upon request.

## References

[1] Davidson E. A., Janssens I. A. (2006). Temperature sensitivity of soil carbon decomposition and feedbacks to climate change. *Nature*.

[2] Ali S., Khan S. M., Siddiq Z. (2022). Carbon sequestration potential of reserve forests present in the protected margalla hills national park. *Journal of King Saud University Science*.

[3] Cheng S. H., Costedoat S., Sterling E. J. (2022). What evidence exists on the links between natural climate solutions and climate change mitigation outcomes in subtropical and tropical terrestrial regions? A systematic map protocol. *Environmental Evidence*.

[4] Houghton R. A., Nassikas A. A. (2017). Global and regional fluxes of carbon from land use and land cover change 1850-2015. *Global Biogeochemical Cycles*.

[5] Gu W., Guo J., Fan K., Chan E. H. W., Lai P. C., Low C. T., Wong P. P. Y. (2016). Dynamic land use change and sustainable urban development in a third-tier city within Yangtze delta. *Proceedings of the International Conference on Geographies of Health and Living in Cities: Making Cities Healthy for All*.

[6] Chen Q., Cai B., Dhakal S. (2017). CO2 emission data for Chinese cities. *Resources, Conservation and Recycling*.

[7] Lang J., Li S., Cheng S. (2018). Chemical characteristics and sources of submicron particles in a city with heavy pollution in China. *Atmosphere*.

[8] Downie A., Lau D., Cowie A., Munroe P. (2014). Approaches to greenhouse gas accounting methods for biomass carbon. *Biomass and Bioenergy*.

[9] Courard-Hauri D., Chancellor R., Rundus A., Boland A. (2016). A method for estimating the current and future carbon content of standing biomass applied to gishwati forest reserve, Rwanda. *Journal of Tropical Forest Science*.

[10] Chen Y., Luo G., Maisupova B. (2016). Carbon budget from forest land use and management in central asia during 1961-2010. *Agricultural and Forest Meteorology*.

[11] Sperow M. (2014). An enhanced method for using the IPCC approach to estimate soil organic carbon storage potential on US agricultural soils. *Agriculture, Ecosystems & Environment*.

[12] Mishra U., Torn M. S., Masanet E., Ogle S. M. (2012). Improving regional soil carbon inventories: combining the IPCC carbon inventory method with regression kriging. *Geoderma*.

[13] Brown M. G., Quinn J. E. (2018). Zoning does not improve the availability of ecosystem services in urban watersheds. A case study from upstate South Carolina, USA. *Ecosystem Services*.

[14] Vizcaino-Bravo Q., Williams-Linera G., Asbjornsen H. (2020). Biodiversity and carbon storage are correlated along a land use intensity gradient in a tropical montane forest watershed, Mexico. *Basic and Applied Ecology*.

[15] Li Y., Liu Z., Li S., Li X. (2022). Multi-scenario simulation analysis of land use and carbon storage changes in changchun city based on FLUS and InVEST model. *Land*.

[16] Choi J., Lee S., Eguchi K., Quanrud D., Takagi H. (2018). An analysis of the carbon fixation change according to the greenbelt deregulation using InVEST model -in case of anyang and gwacheon city-. *Proceedings of the 8th International Conference on Environment Science and Engineering (Icese 2018)*.

[17] Lyu R., Mi L., Zhang J., Xu M., Li J. (2019). Modeling the effects of urban expansion on regional carbon storage by coupling SLEUTH-3r model and InVEST model. *Ecological Research*.

[18] Li K., Cao J., Adamowski J. F. (2021). Assessing the effects of ecological engineering on spatiotemporal dynamics of carbon storage from 2000 to 2016 in the loess plateau area using the InVEST model: a case study in huining county, China. *Environmental Development*.

[19] Yin C., Meng F., Yang X. (2022). Spatio-temporal evolution of urban built-up areas and analysis of driving factors -A comparison of typical cities in north and south China. *Land Use Policy*.

[20] Ma S., Zhao Y., Tan X. (2020). Exploring smart growth boundaries of urban agglomeration with land use spatial optimization: a case study of changsha-zhuzhou-xiangtan city group, China. *Chinese Geographical Science*.

[21] Yang X., Blagodatsky S., Lippe M. (2016). Land-use change impact on time-averaged carbon balances: rubber expansion and reforestation in a biosphere reserve, south-west China. *Forest Ecology and Management*.

[22] Ahirwal J., Gogoi A., Sahoo U. K. (2022). Stability of soil organic carbon pools affected by land use and land cover changes in forests of eastern himalayan region, India. *Catena*.

[23] Chang X., Xing Y., Wang J., Yang H., Gong W. (2022). Effects of land use and cover change (LUCC) on terrestrial carbon stocks in China between 2000 and 2018. *Resources, Conservation and Recycling*.

[24] Li Y., Liu W., Feng Q., Zhu M., Yang L., Zhang J. (2022). Effects of land use and land cover change on soil organic carbon storage in the hexi regions, northwest China. *Journal of Environmental Management*.

[25] Fitts L. A., Russell M. B., Domke G. M., Knight J. K. (2021). Modeling land use change and forest carbon stock changes in temperate forests in the United States. *Carbon Balance and Management*.

[26] Liu Q., Yang D., Cao L., Anderson B. (2022). Assessment and prediction of carbon storage based on land use/land cover dynamics in the tropics: a case study of hainan island, China. *Land*.

[27] Japelaghi M., Hajian F., Gholamalifard M., Pradhan B., Maulud K. N. A., Park H.-J. (2022). Modelling the impact of land cover changes on carbon storage and sequestration in the central zagros region, Iran using ecosystem services approach. *Land*.

[28] Breiman L. (2001). Random forests. *Machine Learning*.

[29] Salem M., El, Mossad M., Mahanna H. (2022). Random forest modelling and evaluation of the performance of a full-scale subsurface constructed wetland plant in Egypt. *Ain Shams Engineering Journal*.

[30] Belgiu M., Dragut L. (2016). Random forest in remote sensing: a review of applications and future directions. *ISPRS Journal of Photogrammetry and Remote Sensing*.

[31] Tang Z., Mei Z., Liu W., Xia Y. (2020). Identification of the key factors affecting Chinese carbon intensity and their historical trends using random forest algorithm. *Journal of Geographical Sciences*.

[32] Dai L., Ge J., Wang L. (2022). Influence of soil properties, topography, and land cover on soil organic carbon and total nitrogen concentration: a case study in qinghai-tibet plateau based on random forest regression and structural equation modeling. *Science of the Total Environment*.

[33] Tirink C. Comparison of bayesian regularized neural network, random forest regression, support vector regression and multivariate adaptive regression splines algorithms to predict body weight from biometrical measurements in thalli sheep. *Kafkas Univ. Vet. Fak. Derg.*.

[34] Yokoyama A., Yamaguchi N. (2020). Comparison between ANN and random forest for leakage current alarm prediction. *Energy Reports*.

[35] Fan P. (2022). Random forest algorithm based on speech for early identification of Parkinson’s disease. *Computational Intelligence and Neuroscience*.

[36] Li L., Levine R. A., Fan J. (2022). Causal effect random forest of interaction trees for learning individualized treatment regimes with multiple treatments in observational studies. *Stat*.

[37] Almaskati N. (2022). The determinants of bank profitability and risk: a random forest approach. *Cogent Economics & Finance*.

[38] Li C., Li L., Zheng J. (2022). China’s public firms’ attitudes towards environmental protection based on sentiment analysis and random forest models. *Sustainability*.

[39] Nofrizal A. Y., Sonobe R., Hiroto Y., Morita A., Ikka T. (2022). Estimating chlorophyll content of zizania latifolia with hyperspectral data and random forest. *International Journal of Electronic Governance*.

[40] Tang K., Zhu H., Ni P. (2021). Spatial downscaling of land surface temperature over heterogeneous regions using random forest regression considering spatial features. *Remote Sensing*.

[41] Zhang M., You W., Qin Q. (2022). Investigation of typical residential block typologies and their impact on pedestrian- level microclimate in summers in nanjing, China. *Frontiers of Architectural Research*.

[42] Zhang M., Dong S., Cheng H., Li F. (2021). Spatio-temporal evolution of urban thermal environment and its driving factors: case study of nanjing, China. *PLoS One*.

[43] Tang S., Wang L. C., Wu X. G. (2019). Valuation of wetland ecosystem services in rapidly urbanizing region: a case study of the nanjing jiangbei new area, China. *Applied Ecology and Environmental Research*.

[44] Liang F., Mao B. (2019). Influencing factors of carbon reserve in natural ecosystem under spatial-temporal dynamic change. *Ekoloji*.

[45] Liu Y., Zhu Y. (2020). Land ecosystem in Yangtze River delta based on InVEST model study on the change of carbon sequestration characteristics (in Chinese). *JOURNAL OF NANJING XIAOZHUANG UNIVERSITY*.

[46] Yan J., Zhang Z., Ding W., Li F. (2014). *Cost-Effectiveness of Rut Treatments for Semi-Rigid Base Asphalt Pavement*.

[47] Yu W., Shi J., Fang Y. (2022). Exploration of urbanization characteristics and their effect on the urban thermal environment in chengdu, China. *Building and Environment*.

[48] Yang S., Lu J., Feng D., Liu F. (2022). Can government-led civilized city construction promote green innovation? Evidence from China. *Environmental Science and Pollution Research International*.

[49] Tao P., Shen H., Zhang Y., Ren P., Zhao J., Jia Y. Status forecast and fault classification of smart meters using LightGBM algorithm improved by random forest. *Wireless Communications and Mobile Computing*.

[50] Li L., Mao C., Sun H., Yuan Y., Lei B. (2020). Digital twin driven green performance evaluation methodology of intelligent manufacturing: hybrid model based on fuzzy rough-sets AHP, multistage weight synthesis, and PROMETHEE II. *Complexity*.

[51] Li W. (2022). Optimization and Application of Random Forest Algorithm for Applied Mathematics Specialty. *Security and Communication Networks*.

[52] Li R., Zhang W., Shen S. (2021). An intelligent heartbeat classification system based on attributable features with AdaBoost+Random forest algorithm. *Journal of Healthcare Engineering*.

[53] Li L., Qu T., Liu Y. (2020). Sustainability assessment of intelligent manufacturing supported by digital twin. *IEEE Access*.

[54] Fan P. (2022). Random Forest Algorithm Based on Speech for Early Identification of Parkinson’s Disease. *Computational Intelligence and Neuroscience*.

[55] Li L., Mao C. (2020). Big data supported PSS evaluation decision in service-oriented manufacturing. *IEEE Access*.

[56] Jiang M., Wang (2021). Xuexia. Research on Intelligent Prediction Method of Financial Crisis of Listed Enterprises Based on Random Forest Algorithm. *Security and Communication Networks*.

[57] Li L., Lei B., Mao C. (January 2022). Digital twin in smart manufacturing. *Journal of Industrial Information Integration*.

[58] Xie H., Dong J., Deng Y., Dai (2022). Yiwen. Prediction Model of the Slope Angle of Rocky Slope Stability Based on Random Forest Algorithm. *Mathematical Problems in Engineering*.

